This article has been retracted.

# Long noncoding RNA BBOX1-AS1 promotes the progression of gastric cancer by regulating the miR-361-3p/Mucin 13 signaling axis

**DOI:** 10.1080/21655979.2022.2072629

**Published:** 2022-06-05

**Authors:** Tao Cai, Binyu Peng, Jun Hu, Yan He

**Affiliations:** a Department of Gastrointestinal Surgery, Hubei No. 3 People’s Hospital of Jianghan University, Wuhan, Hubei, China; b Department of Thyroid and Breast Surgery, Hubei No. 3 People’s Hospital of Jianghan University, Wuhan, Hubei, China

**Keywords:** Gastric cancer, progression, long noncoding RNA, microRNA

## Abstract

Gastric cancer (GC) places a heavy burden on global health, and the information on the molecular mechanism of the progression of GC is still inadequate. Long noncoding RNA (LncRNA) has been confirmed to be widely involved in regulating the progression of GC. Our aim in this study was to explore the role and potential regulatory mechanism of lncRNA BBOX1-AS1 in GC. The expression levels of BBOX1-AS1, miR-361-3p, and MUC13 in GC tissues and cells were evaluated using quantitative real-time polymerase chain reaction and western blotting. The silencer of BBOX1 antisense RNA 1 (BBOX1-AS1) and mucin 13 (MUC13), the mimics and inhibitor of miR-361-3p, and their negative controls were used to alter the expression of these genes. Luciferase reporter, pull-down, and RNA immunoprecipitation assays were performed to verify the correlation between miR-361-3p, BBOX1-AS1, and MUC13. GC cell proliferation, invasion, and apoptosis were detected by cell counting kit-8, transwell, and flow cytometry assays, respectively. An *in vivo* functional experiment was performed to assess the effect of BBOX1-AS1 on GC. The results showed that BBOX1-AS1 was significantly upregulated in GC tissues. Silencing of BBOX1-AS1 inhibited GC cell proliferation and invasion and inhibited tumor growth *in vivo*, whereas it promoted apoptosis. MiR-361-3p was significantly downregulated in GC and counteracted the inhibitory effects of BBOX1-AS1 on GC progression. MUC13, which is targeted by miR-361-3p, is significantly upregulated in GC. MUC13 silencing inhibited GC progression was aborgated by miR-361-3p inhibitor. Collectively, BBOX1-AS1 silencing inhibits GC progression by regulating the miR-361-3p/MUC13 axis, providing a potential therapeutic biomarker for GC.

## Highlights

- LncRNA BBOX1-AS1 sponged miR-361-3p and negatively regulated the expression of miR-361-3p in GC.
- MiR-361-3p directly targeted MUC13 and negatively regulated the expression of MUC13 in GC.
- Silencing lncRNA BBOX1-AS1 suppressed the GC progression via targeting miR-361-3p and inhibiting MUC13 expression.

## 1. Introduction

Gastric cancer (GC) is a global health problem that leads to substantial cancer-related death worldwide[1]. It typically occurs in older individuals. Over the past five decades, the worldwide incidence and mortality due to GC have declined [2]. However, the occurrence of GC varies extensively with geographical location, with half of the new cases occurring in developing countries [3]. High-risk incidences are still being reported in regions such as Eastern Europe, East Asia, and South and Central America. According to incomplete statistics, early tumor resection can result in 5-year survival rates of approximately 90%, and the 5-year survival of patients with advanced GC varies from approximately 20% [3]. Although there are many studies on molecular therapy for GC pathogenesis [4,5], early diagnosis and consecutive early tumor resection are still the leading reasons for the high survival rate of patients with GC [3]. Therefore, a comprehensive understanding of the molecular mechanisms underlying GC is essential.

Long noncoding RNAs (lncRNAs), over 200 nucleotides in length, play critical roles in cancer cell differentiation and epigenetics and have been one of the research hotspots in recent decades. In GC, lncRNAs are regulated at transcriptional and posttranscriptional levels. It affects the progression of GC in several ways. For example, lncRNAs such as maternally expressed 3, H19, and tumor suppressor candidate 7 (TUSC7) have been indicated to be actively involved in the regulation of the GC cell cycle, proliferation, invasion, migration, apoptosis, and tumorigenicity [6–9]. LncRNA BBOX1-AS1 is a new class of lncRNA that has been shown to play a tumor-promoting role, that is, as an oncogenic factor in most tumors. For example, in nasopharyngeal carcinoma, BBOX1-AS1 accelerates tumor cell proliferation and metastasis by regulating miR-3940-3p [10]. In colorectal cancer, BBOX1-AS1 functions as an oncogene to facilitate the tumor malignant phenotype by regulating the miR-361-3p/SH2B1 axis [11]. However, the specific role and regulatory mechanism of BBOX1-AS1 in GC remains unclear.

Accumulating evidence suggests that the interaction between lncRNAs and miRNAs plays a vital role in the occurrence and development of tumors [12]. LncRNAs with targeted binding sites could affect miRNA expression by acting as competitive endogenous RNAs, and then alleviate the inhibitory effects of miRNAs on target gene expression [13,14]. For instance, Xu *et al*. reported that overexpression of lncRNA TINCRL, in GC, induced by the eukaryotic transcription factor SP1 could promote GC cell growth by modulating the steady-state mRNA levels of KLF2 [15]. In addition, lncRNA MT1JP directly targeted miR-214-3p to inhibit the growth of GC cells *in vivo* and *in vitro* [16]. Studies have shown that miR-361-3p, as a tumor suppressor gene, plays an important regulatory role in thyroid cancer [17], prostate cancer, [18] and clear cell renal cell carcinoma [19]. Notably, miR-361-3p is highly expressed in GC, and miR-361-3p effectively reduces the malignant phenotype of GC cells by inhibiting the Wnt/β-catenin pathway [20]. However, the specific mechanisms of miR-361-3p in GC, especially its upstream lncRNAs, require further study.

In recent years, the lncRNA/miRNA/mRNA competing endogenous RNA (ceRNA) network has been reported to regulate GC progression [21]. For instance, lncRNA MAGI2-AS3 promotes GC progression via miR-141/200a/bromodomain containing 4 [22]. In addition, lncRNA HULC can modulate GC progression via the miR-9-5p/myosin heavy chain 9 axis [23]. MUC13, a relatively high-molecular-weight glycoprotein secreted by mucosal tissue, has been shown to promote the development of various tumors, including ovarian cancer [24] and colorectal cancer [25], by regulating numerous signaling pathways. Shimamura *et al*. confirmed that MUC13 expression in GC was significantly higher than that in adjacent normal tissues and that the expression level of MUC13 was closely related to intestinal-type GC (according to Lauren’s classification) [26]. These results suggest that MUC13 plays an important role in promoting GC growth. However, the specific biological functions of MUC13 and MUC13 related ceRNA regulatory networks in GC have not yet been fully elucidated.

In general, we speculate that BBOX1-AS1 may play a pro-oncogenic role in GC by regulating the miR-361-3p/MUC13 pathway. Therefore, our aim in this study is to clarify the specific role of BBOX1-AS1 in GC and its downstream regulatory mechanism. These data provide a new regulatory network for GC progression and suggest a potential therapeutic target for GC.

## 2. Materials and methods

### 2.1 Clinical specimens

A total of 40 human GC tissues and corresponding 40 paracancerous tissues were collected from patients with GC who underwent surgical resection at Hubei No. 3 People’s Hospital of Jianghan University from 2019 to 2020. These patients did not receive radiotherapy or chemotherapy before surgery. Following collection, each sample was confirmed by pathological diagnosis. All the patients provided written informed consent. This study was approved by the Ethics Committee of the Hubei No. 3 People’s Hospital of Jianghan University (Approval No. 2019(015)). The clinical and pathological features of the patients with GC are shown in Table 1.

**Table 1.** Association between BBOX1-AS1 expression and clinicopathological features of gastric cancer

Characteristic	Number (n = 40)	BBOX1-AS1 expression		*P*
		Low	High	
Ago (years)				0.719
< 60	22	12	10	
≥ 60	18	7	11	
Gender				0.425
Male	19	11	8	
Female	21	8	13	
Tumor size (cm)				0.822
< 5	27	13	14	
≥ 5	13	6	7	
Lymph node metastasis				0.031
No	23	16	7	
Yes	17	3	14	
Depth of invasion				0.396
T1 + T2	16	9	7	
T3 + T4	24	10	14	
TNM stage				0.271
I + II	21	10	11	
III + IV	19	9	10	

### 2.2 Cell culture and transfection

One normal gastric epithelial cell line (GES-1) and three GC cell lines (HGC-27, AGS, and GTL-16) were obtained from ATCC (Manassas, VA, USA). The cells were cultured in RPMI-1640 medium (Gibco, USA) supplemented with 10% fetal bovine serum (FBS; Thermo Fisher, Waltham, USA) and 1% penicillin/streptomycin (Gibco, USA) in an incubator (5% CO_2_ and 37°C). After passage, cells in the logarithmic phase were used for the follow-up experimental study.

LncRNA BBOX1-AS1/MUC13 silencers, miR-361-3p inhibitor/mimics, and their corresponding negative controls (NCs) were provided by RiboBio (China). The plasmids were transfected into cells using lipofectamine 2000 according to the manufacturer’s instructions (Invitrogen, USA). Transfection efficiency was determined by quantitative real-time polymerase chain reaction (qRT-PCR) or western blotting 48 h after transfection. Transfection analysis was performed for the following groups: silencer NC (si-NC), BBOX1-AS1 (si-lnc), and MUC13 (si-MUC13); inhibitors of NC (inhibitor-NC) and miR-361-3p (inhibitor); silencer BBOX1-AS1 and miR-361-3p inhibitor (si-lnc+inhibitor); and silencer MUC13 and miR-361-3p inhibitor (si-MUC13+inhibitor).

### 2.3 Cell progression analysis

GC cell proliferation, invasion, and apoptosis were assessed using cell counting kit-8 (CCK-8), transwell, and flow cytometry assays, respectively.

Cell proliferation assay was performed as previously described [27]. Approximately 100 μl transfected cells were seeded into 96-well plates at a density of 1 × 10^4^ cells per well and then incubated at 37°C with 5% CO_2_ for 24, 48, and 72 h, respectively. Then, 10 μl of CCK-8 solution was added to each well and the cells were incubated for another 2 h. Cell viability was detected by measuring the OD_450nm_ using a microplate reader (BioTek, USA).

Cell invasion assay was performed as previously described [28]. Matrigel (Corning, NY, USA) was melted at 4°C overnight and diluted to 1 mg/ml on ice. We added 100 μl Matrigel to the upper chamber with 300 μl of non-serum RPMI-1640 medium and incubated them at 37°C for 5 h. The lower chamber was filled with 500 μl RPMI-1640 medium containing 20% FBS and incubated at 37°C for 24 h. After incubation, the transwell was washed three times with phosphate-buffered saline (PBS), fixed with glutaraldehyde for 15 min, and stained with 0.1% crystal violet for 20 min. Twenty minutes later, five visuals were randomly selected and invasive cells were counted under a 400× inverted microscope (Olympus X51 Inverted Microscope).

A commercial kit purchased from Vazyme Co. Ltd (#A211-01; Nanjing, China) was used for cell apoptosis analysis according to a previous study [29]. Briefly, the cells were collected, suspended, washed, and stained with annexin V-FITC and PI staining solution. After 10 min of incubation, the number of apoptotic cells was analyzed by flow cytometry using a FACSCalibur flow cytometer (BD Biosciences, USA).

### 2.4 Xenograft mouse model

Short hairpin RNA (shRNA) NC (sh-NC) and BBOX1-AS1 (sh-lnc) were synthesized by GeneBio (Guangzhou, China). Ten BALB/c nude mice (4-week-old, specific pathogen-free degree) were provided by Charles River (Raleigh, USA). These mice were then injected with 5 × 10^5^ sh-lnc (*n* = 5) and sh-NC (*n* = 5) HGC-27 cells. The mice were housed for 5 weeks at room temperature and given water and food *ad libitum*. Mice were euthanized after 5 weeks, and their tumor tissues were isolated, weighed, and measured. Tumor size was measured according to the method described by Digklia *et al*. [30]. Our study has been approved by the Ethics Committee of Hubei No. 3 People’s Hospital of Jianghan University (Wuhan, China). Our study adhered to the requirements and guidelines of the Ethics Committee of Hubei No. 3 People’s Hospital of Jianghan University.

### 2.5 Quantitative real-time PCR analysis

RT-PCR was performed as previously described [31]. Total RNA was extracted from GC cells and tissues using TRIzol® reagent (Invitrogen; Thermo Fisher Scientific, Waltham, MA, USA), according to the manufacturer’s instructions. Primers were synthesized by Synbio Technologies (Suzhou, China). cDNAs were synthesized using a reverse transcription kit (Invitrogen, USA). The one-step SYBR kit obtained from Vazyme (China) was used for PCR and the manufacturer’s instructions were followed. PCR was conducted on an Applied Biosystems 7300 RT-PCR system (Foster City, CA, USA). Relative expression was measured using the 2^−ΔΔCt^ method [32]. GAPDH and U6 were used as internal controls to analyze lncRNA/mRNA and miRNA, respectively. The primers used for BBOX1-AS1, MUC13, miR-361-3p, GAPDH, and U6 are listed in Table 2.

**Table 2.** Sequences of primers used in qRT-PCR

Primer Name:	Sequences (5’ to 3’)
BBOX1-AS1	Forward primer, TGCAACTCCAAACCTAACG
	Reverse primer, GAGTGACTGGGGTCAGGGTA
miR-361-3p	Forward primer, GAGTCCCCCAGGTGTGATTC
	Reverse primer, GTCGTATCCAGTGCGTGTC
MUC13	Forward primer, AGAAACATTC CATGGCCTATCAA
	Reverse primer, TGTCCA TAAACAGATGTGCCAAA
CLDN4	Forward primer, CCAAGTCATGGTGTGCTGAG
	Reverse primer, CACTGGGCTGCTTCTAGGTC
GAPDH	Forward primer, AAT CCCATCACCATCTTCCA
	Reverse primer, TGGACTCCACGACGTACTCA
U6	Forward primer, CTCGCTTCGGCAGCACATATACT
	Reverse primer, ACGCTTCACGAATTTGCGTGTC

### 2.6 Western blot analysis

The total protein was extracted from transfected GC cells using RIPA buffer (Thermo Fisher Scientific). A BCA protein quantification kit (Beyotime, China) was used to determine the protein concentration. Sodium dodecyl sulfate-polyacrylamide gel electrophoresis was performed for protein separation. The gels were transferred to poly (polyvinylidene fluoride) (PVDF) membranes and blocked with 5% nonfat milk for 1 h at room temperature. These membranes were incubated with primary antibodies against GAPDH (1:1,000; #bs-10900 R; Bioss, Beijing, China) and MUC13 (1:1,000; #bs-1,074 R; Bioss, Beijing, China) at 4°C overnight and then incubated with the secondary antibody of horseradish peroxidase‑conjugated goat anti‑rabbit IgG (1:5,000; #ab6721; Abcam) for 1 h at 25°C. Finally, the protein bands were visualized using enhanced chemiluminescence (Pierce, Thermo Fisher Scientific, USA). The grayscale of the protein bands was analyzed using ImageJ software.

### 2.7 Luciferase reporter assay

The wild-type (WT) BBOX1-AS1 or MUC13 3′UTR with binding sites of miR-361-3p or mutated (Mut) BBOX1-AS1 or MUC13 3′UTR without binding sites of miR-361-3p were constructed by Sangon (Shanghai, China). Then, WT and Mut BBOX1-AS1 or MUC13 3′UTR were inserted into the pGL3 vector (Promega, Madison, USA). miR-NC or miR-361-3p mimics were co-transfected into HGC-27 and GTL-16 cells along with WT/Mut-BBOX1-AS1 or WT/Mut-MUC13 for 24 h. Relative luciferase activities were determined using the Dual Luciferase Assay Kit (Promega, USA).

### 2.8 RNA immunoprecipitation assay

The Magna RNA immunoprecipitation (RIP) Kit (Millipore, Bedford, MA) was used for the RIP assay following the manufacturer’s instructions as previously described [33]. Briefly, HGC-27 and GTL-16 cell suspensions were prepared using RIP buffer. Furthermore, Ago2/IgG antibody (Cambridge, MA, USA) conjugated with magnetic beads and cell suspension were incubated overnight at 4°C. The cell suspension was digested with protease K, followed by RNA extraction. The precipitated RNA was analyzed by qRT-PCR.

### 2.9 RNA pull-down assay

A biotin-labeled miRNA pull-down assay was performed to verify the connection between miR-361-3p and MUC13, as previously described [34]. Briefly, the HGC-27 and GTL-16 cells were washed with PBS and harvested using a cell scraper. These cells were then incubated with 0.5 mL of 70 mM KCl, 25 mM Tris-HCl (pH 7.5), 0.05% NP-40, 2.5 mM EDTA, and 80 U/mL RNase inhibitor on ice for 25 min. The supernatant containing mRNA was obtained after centrifugation at 4°C, 12000 × *g*, 15 min. Subsequently, biotinylated miR-361-3p (Bio-miR-361-3p) and the corresponding negative control (Bio-NC) were added to the supernatant and incubated with streptavidin Mutein Matrix (Roche) and an extraction buffer for 3 h. Biotinylated RNAs/mRNAs were washed and detected using qRT-PCR.

### 2.10 Bioinformatic analysis

The binding sites of miR-361-3p on MUC13, BBOX1-AS1, and CLDN4 were predicted using StarBase v2.0 (http://starbase.sysu.edu.cn/starbase2). The expression levels of BBOX1-AS1, MUC13, and miR-361-3p were downloaded in GEPIA (http://gepia.cancer-pku.cn/). The target genes were predicted using ENCORI (http://starbase.sysu.edu.cn/) and TargetScan v7.2 (http://www.targetscan.org/vert_72/).

### 2.11 Statistical analysis

GraphPad Prism 8.0 (San Diego, CA, USA) was utilized for data processing and drawing graphs. All data were exhibited as mean ± standard deviation. Student’s *t*-test or one-way ANOVA was conducted to determine significant differences between two groups or among multiple groups. Pearson analysis was done to find the expression level between miR-361-3p and BBOX1-AS1 or MUC13. *P* < 0.05 was deemed statistically significant.

## 3. Results

The purpose of this study was to explore the specific role of BBOX1-AS1 in GC and its underlying downstream regulatory pathways. In this study, we first detected the expression of BBOX1-AS1, miR-361-3p, and MUC13 in GC tissues and cells. Furthermore, the expression of BBOX1-AS1, miR-361-3p, and MUC13 was altered by transfection with siRNA-encoding plasmids and an miR inhibitor. Subsequently, functional experiments with GC cells were performed to detect cell proliferation, invasion, and apoptosis. Finally, we demonstrated that BBOX1-AS1 could upregulate the expression of MUC13 by sponging miR-361-3p, thus promoting GC progression.

### 3.1 BBOX1-AS1 was significantly upregulated in GC

First, we assessed the expression of BBOX1-AS1 in GC samples by qRT-PCR. The expression level of BBOX1-AS predicted by GEPIA was upregulated in the GC samples (*P* < 0.01; Figure 1(a)). Meanwhile, the expression of BBOX1-AS1 in GC tissues (40 cases in total) was higher than that in adjacent normal tissues (*P* < 0.0001; Figure 1(b)). As evaluated *in vitro*, the expression level of BBOX1-AS was higher in GC cells (HGC-27, AGS, and GTL-16) than in GES-1 cells, especially in HGC-27 and GTL-16 cells (*P* < 0.001; Figure 1(c)). Additionally, BBOX1-AS1 was mainly distributed in the cytoplasm (*P* < 0.001; Figure 1(d)), indicating that BBOX1-AS1 may play a role in GC progression via the ceRNA mechanism. These data suggest that the high expression of BBOX1-AS1 may play a pro-oncogenic role in GC.

**Figure 1.** BBOX1-AS1 was significantly upregulated in GC. (a) GEPIA on predicting the expression levels of BBOX1-AS1 in GC tissues and normal tissues. (b, c) The expression level of BBOX1-AS1 in GC clinical samples (b) and GC cell lines (c) was detected by qRT-PCR. (d) The distribution of BBOX1-AS1 in cytoplasm and nucleus of HGC-27 and GTL-16 cell lines, using GAPDH and U6 as the references. *P < 0.05, **P < 0.001.

### 3.2 Silenced BBOX1-AS1 inhibited the GC cell proliferation and invasion, promoted apoptosis in vitro, and reduced tumor growth in vivo

Subsequently, we evaluated the role of BBOX1-AS1 in GC progression. We constructed an lncRNA BBOX1-AS1 knockdown plasmid (si-lnc). As shown in Figure 2(a), compared to the si-NC group, the expression of BBOX1-AS1 was markedly decreased in the si-lnc group, indicating that cell silencer transfection was successfully constructed. The effect of BBOX1-AS1 knockdown on GC cell growth *in vitro* was assessed in both HGC-27 and GTL-16 cells. CCK-8 results showed that cell proliferation was significantly reduced in HGC-27 and GTL-16 cells transfected with si-lnc compared to si-NC (*P* < 0.001; Figure 2(b)). Transwell assay results demonstrated that compared with the si-NC group, the number of invasive GC cells was significantly decreased by BBOX1-AS1 knockdown (*P* < 0.001; Figure 2(c)). Moreover, flow cytometric analysis revealed that the apoptosis rate in the si-lnc group was enhanced by 6 folds compared to that in the si-NC group, suggesting that BBOX1-AS1 knockdown significantly accelerated cell apoptosis (*P* < 0.001; Figure 2(d)). *In vivo* xenograft tumor experiments were performed to verify the role of BBOX1-AS1 in GC tumor growth. We found that the tumor volume and weight were significantly decreased in HGC-27 cells transfected with sh-lnc compared to those transfected with sh-NC (*P* < 0.001; Figure 2(e)). Collectively, silencing BBOX1-AS1 significantly repressed GC cell proliferation and invasion, promoted apoptosis *in vitro*, and reduced tumor growth *in vivo*.

**Figure 2.** BBOX1-AS1 inhibited the GC cell proliferation and invasion, promoted apoptosis *in vitro*, and reduced tumor growth *in vivo*. (a) The expression level of BBOX1-AS1 in si-NC and si-lnc groups of HGC-27 and GTL-16 cell lines was evaluated by qRT-PCR. (b) The OD_450nm_ at si-NC and si-lnc groups of HGC-27 and GTL-16 cell lines were evaluated by CCK-8 assay. **P < 0.001 *vs* si-NC. (c) The cell invasion of HGC-27 and GTL-16 cell lines transfected with si-NC and si-lnc was assessed by Transwell assay. Si-NC, silencer negative control; si-lnc, silencer BBOX1-AS1. **P < 0.001 *vs* si-NC. (d) The cell apoptosis of HGC-27 and GTL-16 cell lines transfected with si-NC and si-lnc was assessed by flow cytometry. **P < 0.001 *vs* si-NC. (e) The tumor volume and weight were measured in groups of sh-NC and sh-lnc. Sh-NC, knockdown negative control; sh-lnc, knockdown BBOX1-AS1. **P < 0.001 *vs* sh-NC.

### 3.3 MiR-361-3p was a target for BBOX1-AS1

To study the downstream regulatory pathway of BBOX1-AS1 in GC progression, sponging miRNAs of BBOX1-AS1 were screened. As predicted by StarBase, BBOX1-AS1 has potential binding sites for miR-361-3p (Figure 3(a)). Luciferase reporter and RIP assays were performed to verify the relationship between BBOX1-AS1 and miR-361-3p. Luciferase reporter assay results indicated that miR-361-3p mimics significantly attenuated the luciferase activity of the BBOX1-AS1-WT vector but had no effect on the BBOX1-AS1-Mut vector (*P* < 0.001; Figure 3(b)). The RIP assay results revealed that anti-Ago2 significantly increased the enrichment of BBOX1-AS1 on miR-361-3p (*P* < 0.001; Figure 3(c)). These results revealed that BBOX1-AS1 directly targets miR-361-3p. In addition, expression analysis showed that miR-361-3p expression was significantly lower in GC tissues than in normal tissues (*P* < 0.0001; Figure 3(d)). Compared to GES-1 cells, HGC-27 and GTL-16 cells showed low miR-361-3p expression (*P* < 0.001; Figure 3(e)). Furthermore, a negative correlation was found between BBOX1-AS1 and miR-361-3p mRNA expression levels using Pearson correlation analysis (*R*^2^ = 0.5918, *P* < 0.0001; Figure 3(f)). These results suggested that BBOX-AS1 targeted miR-361-3p and negatively regulated its expression in GC.

**Figure 3.** MiR-361-3p was a target of BBOX1-AS1. (a) StarBase predicted the binding sites of BBOX1-AS1 on miR-361-3p. (b) The luciferase reporter analysis on miR-361-3p and BBOX1-AS1. **P < 0.001 *vs* mimic-NC. (c) RIP analysis on BBOX-AS1 and miR-361-3p. **P < 0.001 *vs* Anti-IgG. (d, e) The expression level of miR-361-3p in GC clinical samples (d) and GC cell lines (e) was detected by qRT-PCR. **P < 0.001. (f) *Pearson* correlation analysis on the relationship between BBOX1-AS1 and miR-361-3p.

### 3.4 MiR-361-3p knockdown counteracted the functional role of BBOX1-AS1 silencing on GC progression

To further investigate the role of BBOX1-AS1 in GC cell growth via regulation of miR-361-3p, we constructed an miR-361-3p knockdown plasmid (inhibitor). The expression of miR-361-3p was measured in the si-NC, inhibitor-NC, inhibitor, si-lnc, and si-lnc + inhibitor groups by qRT-PCR. The results showed that miR-361-3p was significantly upregulated by BBOX1-AS1 silencing and this change was alleviated by the miR-361-3p inhibitor (*P* < 0.05; Figure 4(a)). *In vitro* functional experiments suggested that cell proliferation and invasion were significantly promoted by miR-361-3p knockdown and that these changes were alleviated by BBOX1-AS1 silencing (*P* < 0.001; Figure 4(b,c)). As expected, cell apoptosis was significantly reduced in HGC-27 and GTL-16 cells transfected with miR-361-3p inhibitor, but this inhibitory effect of apoptosis induced by miR-361-3p downregulation was reversed in GC cells transfected with miR-361-3p inhibitor and si-lnc (*P* < 0.001; Figure 4(d)). BBOX1-AS1 silencer and miR-361-3p inhibitor have opposing functions in promoting GC progression. In summary, silencing of BBOX1-AS1 inhibited GC progression by sponging miR-361-3p.

**Figure 4.** MiR-361-3p knockdown counteracted the functional role of BBOX1-AS1 silencing on GC progression. (a) The expression level of miR-361-3p was evaluated in groups of si-NC, inhibitor-NC, inhibitor, si-lnc, and si-lnc+inhibitor by qRT-PCR. (b-d) The cell proliferation (b), invasion (c), and apoptosis (d) were measured in groups of si-NC, inhibitor-NC, inhibitor, si-lnc, and si-lnc+inhibitor using CCK-8, Transwell and flow cytometry assays, respectively. **P < 0.001 *vs* si-NC, ^&&^*P* < 0.001 vs inhibitor-NC. ^##^*P* < 0.001 *vs* si-lnc+inhibitor.

### 3.5 *MUC13* was targeted by miR-361-3p

We characterized the downstream target genes of miR-361-3p. Target genes of miR-361-3p were screened and verified using GEPIA and ENCORI. MUC13 and CLDN4 were found at the intersection of the gene sets (Figure 5(a)). RNA pull-down assay results showed that MUC13 exhibited higher enrichment than CLDN4 on miR-361-3p (*P* < 0.001; Figure 5(b)). The ENCORI database revealed complementary sequence sites between miR-361-3p and BBOX1-AS1 (Figure 5(c)). Luciferase reporter assay results showed that the miR-361-3p mimic strongly reduced luciferase activity in HGC-27 and GTL-16 cells introduced with MUC13-WT but not the MUC13-MUT vector (*P* < 0.001; Figure 5(d)). Expression analysis demonstrated that MUC13 expression was higher in HGC-27 and GTL-16 cells than in GES-1 cells (*P* < 0.001; Figure 5(e)). Similarly, MUC13 expression was upregulated in GC tissues compared to that in normal tissues (*P* < 0.001; Figure 5(f)). Pearson’s analysis revealed an opposed expression trend between miR-361-3p and MUC13 (*R*^2^ = 0.5748, *P* < 0.0001; Figure 5(g)). These data validated that MUC13 was targeted by miR-361-3p.

**Figure 5.** MUC13 was targeted by miR-361-3p. (a) MUC13 and CLDN4 were predicted and screened as the target genes of miR-361-3p using GEPIA and ENCORI. (b) RNA pull-down analysis on the interaction between MUC13 and CLDN4 of miR-361-3p. **P < 0.001 *vs* Bio-NC. (c) The binding sites of MUC13 on miR-361-3p were predicted by StarBase. (d) The luciferase reporter analysis on the relationship between miR-361-3p and MUC13. **P < 0.001 *vs* miR-NC. (e, f) The expression level of MUC13 in GC clinical samples (e) and GC cell lines (f) was detected by qRT-PCR.  (g) *Pearson* analysis revealed the expression relationship between miR-361-3p and MUC13.

### 3.6 MiR-361-3p knockdown promoted GC progression by targeting MUC13

Based on previous results, we speculated that miR-361-3p could affect GC cell growth by regulating MUC13 expression. Western blotting showed that the expression of MUC13 was significantly reduced in HGC-27 and GTL-16 cells transfected with alone si-MUC13, and MUC13 expression inhibited by si-MUC13 was partially relieved by an additional miR-361-3p inhibitor, demonstrating the successful transfection of siRNA for MUC13 (*P* < 0.001; Figure 6(a)). CCK-8 and transwell assays revealed that MUC13 knockdown substantially inhibited the proliferation and invasion of HGC-27 and GTL-16 cells. GC cell proliferation and invasion abilities blocked by low MUC13 expression were partly alleviated by the miR-361-3p inhibitor (*P* < 0.001; Figure 6(b,c)). As expected, the flow cytometry assay showed that GC cell apoptosis could be promoted by MUC13 knockdown but repressed by the miR-361-3p inhibitor. Apoptosis induced by MUC13 knockdown was partially inhibited by the miR-361-3p inhibitor (*P* < 0.001; Figure 6(d)). In summary, overexpression of BBOX1-AS1 promotes GC progression by regulating the MUC13/miR-361-3p axis.

**Figure 6.** MiR-361-3p knockdown promoted GC progression by targeting MUC13. (a) The expression level of miR-361-3p was evaluated in groups of si-NC, inhibitor-NC, inhibitor, si-MUC13, and si-MUC13+ inhibitor by qRT-PCR. (b-d) The cell proliferation (b), invasion (c), and apoptosis (d) were measured in groups of si-NC, inhibitor-NC, inhibitor, si-MUC13, and si-MUC13+ inhibitor using CCK-8, Transwell and flow cytometry assays, respectively. **P < 0.001 *vs* si-NC, ^&&^*P* < 0.001 *vs* inhibitor-NC. ^##^*P* < 0.001 *vs* si-lnc+inhibitor.

## 4. Discussion

GC is a worldwide health issue, with a 5-year survival rate of less than 10% when patients are diagnosed at an advanced stage, but the rate is 85% if the patients are detected at an earlier stage [35]. Therefore, in-depth studies of the molecular mechanisms of GC are critical. Several studies have shown that lncRNAs play critical roles in GC progression [22,36]. However, the role of BBOX1-AS1 in GC remains unclear. We investigated the function of BBOX1-AS1 in GC progression and found that BBOX1-AS1 was significantly upregulated in GC. Moreover, BBOX1-AS1 silencing inhibited the progression of GC. Additionally, BBOX1-AS1 knockdown inhibited GC progression by regulating the miR-361-3p/MUC13 axis.

BBOX1-AS1 has been reported to play a role in several cancers [11,37–40]. In line with the findings of our present study, Xu *et al*. [37] demonstrated that the downregulation of BBOX1-AS1 inhibited the growth and migration of cervical cancer cells. BBOX1-AS1 is also upregulated in colorectal cancer cell lines, and knockdown of BBOX1-AS1 can enhance cell progression [11]. Moreover, BBOX1-AS1 was upregulated in lung cancer tissues, and BBOX1-AS1 deficiency inhibited cell proliferation, migration, and invasion [39]. Notably, BBOX1-AS1 was also found to be upregulated in GC, as reported by Yang *et al*. [40], which indicated that the downregulation of BBOX1-AS1 effectively inhibited GC cell proliferation and promoted cell apoptosis. This observation is in agreement with the results of the present study. Compared to GES-1 cells, BBOX1-AS1 was upregulated in three GC cell lines (HGC-27, AGS, and GTL-16). Furthermore, we conducted a more comprehensive analysis of the role of BBOX1-AS1 in GC progression *in vitro* and *in vivo*. Silencing of BBOX1-AS1 reduced cell proliferation and invasion while promoting apoptosis.

lncRNAs can sponge a large number of miRNAs and reduce their ability to interfere with their target genes. Therefore, miRNAs act as associate nodes and play an important role. We found that BBOX1-AS1 was mainly distributed in the cytoplasm, suggesting that BBOX1-AS1 may exert a cancer-promoting effect as a ceRNA in GC. Subsequently, we verified that miR-361-3p is sponged by BBOX1-AS1 and exhibits opposing functions. Previous studies have demonstrated a counteracting role of BBOX1-AS1 and miR-361-3p in cervical cancer [37], colorectal cancer [11], and ovarian cancer [38]. The results of these studies are consistent with those of the present study. The inhibitor miR-361-3p and BBOX1-AS1 have opposing functions in promoting GC progression. Xu *et al*. [37] also demonstrated that miR-361-3p reverses the role of BBOX1-AS1 upregulation in cervical cancer progression. Not only sponged by BBOX1-AS1, but miR-361-3p is also sponged by other lncRNAs, such as ABHD11-AS1 [41] and SNHG22 [20], and plays an essential role in GC.

miRNAs function by targeting mRNAs at the posttranscriptional level [42]. In this study, two target genes (MUC13 and CLDN4) of miR-361-3p were selected. Through comparison, we found that MUC13 was more enriched than CLDN4 in RNA pull-down analysis. Luciferase reporter analysis confirmed that miR-361-3p could directly target MUC13. Therefore, MUC13 was selected for further study. None of the previous studies have demonstrated the regulation of miR-361-3p and MUC13. Nevertheless, MUC13 has been widely reported to regulate various cancers, including ovarian cancer [24], colon cancer [25], colorectal cancer [43,44], and gastric cancer [26,45]. MUC13 is typically expressed in the intestine and is correlated with the gastric colon and cancer [26,43,44]. Gupta *et al*. [25] demonstrated that overexpression of MUC13 increases colony formation, cell growth, migration, and invasion in colon cancer. Their results were consistent with those of the present study, in which we demonstrated that MUC13 was significantly upregulated in GC, and overexpressed MUC13 promoted GC progression. Sheng *et al*. [44] demonstrated that MUC13 activates the NF-κB pathway and upregulates the critical apoptosis regulator to protect human colorectal cancer cells from death. Shimamura *et al*. [26] revealed that MUC13 was overexpressed in intestinal-type GC and was a diagnostic and therapeutic target. Their results are consistent with those of our study. Previous studies have reported that overexpressed MUC13 significantly enhances HER2, ERK, and Akt [46]. The present study demonstrated that MUC13 competitively binds miR-361-3p with BBOX1-AS1, which is upregulated in GC, and that overexpression of BBOX1-AS1 promotes cell progression. The final point is worth discussing: In the flow cytometry experiment, both early and late apoptotic cells were calculated as the incidence of apoptotic cell death. The results of this study showed that GC cells were mainly in the early stages of apoptosis, with fewer apoptotic cells in the late stages. We speculate that the regulation of GC cell apoptosis by the BBOX1-AS1/miR-361-3p/MUC13 axis is mainly directed toward early apoptosis.

## 5. Conclusion

We verified the sponging and targeting roles of miR-361-3p in BBOX1-AS1 and MUC13 cells. Moreover, we demonstrated that the overexpression of BBOX1-AS1 promotes GC progression by regulating the miR-361-3p/MUC13 axis. The present study revealed the regulatory mechanism of BBOX1-AS1 and may provide a promising therapeutic strategy for GC.

## Supplementary Material

Supplemental Material

Supplemental Material
